The article "The Black-Box Deconstruction of Dynamic Sustainable Development Ability Driving Environmental Performance of Manufacturing Enterprises" was retracted in 2023. Reasons: signs of a paper mill; suspected computer-generated content; unreliable results or conclusions; concerns about the data.

# The Black-Box Deconstruction of Dynamic Sustainable Development Ability Driving Environmental Performance of Manufacturing Enterprises

**DOI:** 10.1155/2022/1734008

**Published:** 2022-08-24

**Authors:** Qiang Liu, Wanqian Zhang, Ziwei Gao, Wei Yang

**Affiliations:** School of Economics and Management, Liaoning University of Technology, Jinzhou 121001, China

## Abstract

Based on the conceptual model of the black-box deconstruction of dynamic sustainable development ability driving environmental performance of manufacturing enterprises, the nonparametric percentile bootstrap method based on deviation correction is used to demonstrate the theoretical hypothesis and empirically deconstruct the black-box of dynamic sustainable development driving environmental performance. Empirical results show that (1) dynamic sustainable development ability has a positive influence on environmental performance; (2) green resource integration ability, green duality, low-carbon manufacturing practice, and green intelligence capital play mediating roles in the influence of dynamic sustainable development ability on environmental performance; and (3) environmental regulation positively moderates the mediating mechanism of green resource integration ability, green duality, low-carbon manufacturing practice, and green intelligence capital of the relationships between dynamic sustainable development ability and environmental performance.

## 1. Introduction

In the process of rapid economic growth, environmental problems emerge in endlessly, which have posed a great threat to production and life, and have aroused the great attention of the government. In order to prevent environmental problems from getting worse, the CPC Central Committee actively advocated the construction of resource-saving and environment-friendly society in 2007. At the same time, the environmental management awareness of manufacturing enterprises has also been aroused. The concept of green development has gradually become the mainstream. Economic benefits are no longer the only standard to measure the success of the manufacturing enterprise. Under the framework of dynamic sustainable development, the decisions regarding how to respond to the trend, implement the concept of green development, enhance the ability of green management, and finally obtain good environmental performance are the main key problems to be solved urgently in the academic and industrial circles. Some scholars had studied the relationships between sustainable development ability and value creation, or the relationships between green management and environmental performance, and had obtained relevant research results with reference and inspiration [1–52]. However, few scholars had taken manufacturing enterprises as the objects of empirical analysis to conduct empirical research on the influence mechanism of dynamic sustainable development ability on environmental performance and carry out empirical deconstruction of the black-box of environmental performance driven by dynamic sustainable development ability of manufacturing enterprises. The general meaning of the black-box of dynamic sustainable development ability driving environmental performance of manufacturing enterprises refers to the influence mechanism of dynamic sustainable development ability on environmental performance of manufacturing enterprises. In view of the reasoning process, based on the background of green leading development, this study will deeply deconstruct the black-box of dynamic sustainable development ability driving environmental performance of manufacturing enterprises, improve and enrich the theoretical framework and conceptual model of the black-box of dynamic sustainable development ability driving environmental performance of manufacturing enterprises, explore the influence mechanism of dynamic sustainable development ability on environmental performance of manufacturing enterprises under the action of different situational variables, analyze the effectiveness of various mediating variables and boundary conditions, and pry the black-box of green development of manufacturing enterprises. The research results will have important theoretical reference and practical management enlightenment for guiding manufacturing enterprises to effectively implement the sustainable development framework and complete the bilateral transformation. The research results will also provide a practical basis and quantitative foundation for advocating environmental management awareness, promoting dynamic sustainable development ability, and enhancing environmental performance of manufacturing enterprises with the help of mediating variables and moderating variables.

## 2. Conceptual Model

### 2.1. Theoretical Hypothesis

#### 2.1.1. Direct Relationships between Dynamic Sustainable Development Ability and Environmental Performance

The dynamic sustainable development ability of the manufacturing enterprise refers to the ability of the manufacturing enterprise to identify problems and opportunities, and achieve the goals by dynamically adjusting its own resources [2, 46–48]. Sustainable development ability refers to the ability of the manufacturing enterprise to achieve the performance objectives on the premise of avoiding or reducing pollution and damage to the environment [1]. Teece and Wijethilake defined dynamic ability as the ability of manufacturing enterprises to maintain and enhance market competitiveness by moderating their own resources [46, 47]. Based on the research results, scholars Shang et al. integrated the sustainable development ability and dynamic ability to obtain the sustainable development ability of manufacturing enterprises, and believed that combining the two sections and components is the key path for manufacturing enterprises to avoid or reduce the interference of various uncertain factors in their growth process and adapt to the new-normal environments and circumstances [2, 4, 5].

If the manufacturing enterprise wants to occupy the more favorable position in the market and obtain more resources, dynamic sustainable development ability is an indispensable and crucial factor [6]. Philip [8] believed that sustainable development ability included two levels (increasing enterprise performance and market share), and there was a positive correlation between sustainable development ability and shareholders' recognition of the manufacturing enterprise. Improving the dynamic sustainable development ability of manufacturing enterprises, driving the further accumulation of accumulated resources, triggering manufacturing enterprises to improve their market competitiveness and market share, increasing profits, expanding scale, and promoting the dynamic sustainable development ability can have a positive effect on environmental performance [1–9]. At the same time, many scholars in related fields had believed that under the framework of sustainable development, the manufacturing enterprise performance should be evaluated from the environmental benefits, social benefits, and other aspects [1–12]. Based on the above research results, this study believes that the dynamic sustainable development ability is the key factor for manufacturing enterprises to achieve higher environmental performance. Therefore, this paper proposes the following hypothesis:

  H1: dynamic sustainable development ability has a significant positive influence on environmental performance of manufacturing enterprises.

#### 2.1.2. Mediating Roles

*(1) The Mediating Role of Green Resource Integration Ability*. Green resource integration ability is the ability of the manufacturing enterprise to further optimize the original resource structure system, establish the new green resource system, and identify and deal with the corresponding internal and external resources on the premise of obtaining the external resources and requirements according to the connotation and requirements of sustainable development [13–15]. Green resources are mostly in a disorderly and chaotic state before being developed and integrated. In order to make manufacturing enterprises obtain more and better environmental benefits, it is necessary to scientifically deal with the fragmented resources, and make a strong sense of fusing and integrating the fragmented resources into organization value, so as to promote them to give full play to their use value. Identifying, absorbing, allocating, and integrating the internal and external green resources of the manufacturing enterprise are the four basic processes for the manufacturing enterprise to improve the green resource integration ability. Among them, the identifying ability of green resources can help manufacturing enterprises better and faster tap the key resources needed for their development, which plays a major role in improving environmental performance. The ability to absorb green resources can help manufacturing enterprises quickly absorb the green resources in the external environment that they need, which plays the role in promoting manufacturing enterprises to obtain high benefits. The ability to allocate green resources plays an important role in the efficient use of existing resources. The integration ability of green resources is an indispensable driving force for manufacturing enterprises to create and give play to green values. The higher the efficiency of resource utilization and integration, the better the environmental benefits of manufacturing enterprises and the higher the environmental performance [13, 15]. Dynamic sustainable development ability needs to identify, adjust, and integrate their own resources with the help of green resource integration ability, so as to feed back the dynamic sustainable development ability of manufacturing enterprises; that is, green resource integration ability is the key channel for manufacturing enterprises to give full play to the dynamic sustainable development ability. Therefore, based on the above analysis, the following theoretical hypothesis is put forward:

  H2: green resource integration ability plays a mediating role in the process of the influence of dynamic sustainable development ability on environmental performance; that is, dynamic sustainable development ability indirectly affects environmental performance by influencing green resource integration ability.

*(2) The Mediating Role of Green Duality*. Duality refers to the fact that the influence of constituent elements or influencing factors on something is equal or equal in two aspects. It is believed that the influencing factors or constituent elements do not act and affect things unilaterally, but the joint actions between the influencing factors or constituent elements affect things [16]. Many scholars had interpreted the concept of duality from different perspectives. Cao et al. [18] conceptualized the term duality and decomposed it into a two-dimensional composite structure, including the balance dimension and the interaction dimension. Since then, some scholars had further analyzed and explored the concept of duality, further defined and improved the concept of balance degree, and put forward the concept of organic balance [19]. Lin et al. [20] believed that if Chinese manufacturing enterprises wanted to improve the innovation performance, they should make the balance between the two dimensions of quality management practice (exploration dimension and utilization dimension) according to the characteristics of internal and external environment and resources, and reduce or even avoid the probability of competing for limited resources during the implementation of the two dimensions of quality management practice, so as to make the two dimensions complement each other. Lin et al. [20] analyzed the balance dimensions of duality; the relationships between interaction dimension and enterprise innovation performance are deeply studied. Green duality refers to green exploration and green utilization. Under the framework of dynamic sustainable development ability, green exploration focuses on the development and design of new concepts, and adopts innovative solutions that break the habitual way of thinking to solve environmental problems. Compared with green exploration, green utilization focuses more on introducing existing and well-developed technologies, or improving the existing production processes and products of the manufacturing enterprise, so as to significantly improve the resource utilization rate of the manufacturing enterprise and effectively reduce the damage and pollution caused by the manufacturing enterprise to the environment [16]. No matter what angle, green duality can have a significant positive influence on environmental performance. At the same time, the strong dynamic sustainable development ability of the manufacturing enterprise means that the manufacturing enterprise is sensitive to environmental changes and has a strong ability to adjust its own resources, which provides a strong support for the manufacturing enterprise to find out innovation points and continuously render the resources required for innovation. Whether it is breakthrough innovation or sublimation innovation on its own basis, green duality will magnify the influence of dynamic sustainable development ability on environmental performance. In addition, in order to better study the influence mechanism of green exploration and green utilization on environmental performance, the concepts of green exploration and green utilization in duality are introduced into green innovation practice by referring to and drawing on relevant research results [16], and green exploration *x* and green utilization *y* are organically combined to study green duality from the balance and interaction dimensions. Referring to the existing achievements, the mathematical expression *x* × *y* reflects the interaction dimension of green exploration and green utilization [18]. The mathematical expression 1 − |*x* − *y*|/(*x*+*y*) represents the balance dimension of green exploration and green utilization [18]. Based on the above analysis, this paper puts forward the following theoretical hypotheses:

  H3: green duality plays a mediating role in the process of the influence of dynamic sustainable development ability on environmental performance; that is, dynamic sustainable development ability indirectly affects environmental performance by influencing green duality.
  H3a: green dual interaction dimension plays a mediating role in the process of the influence of dynamic sustainable development ability on environmental performance; that is, dynamic sustainable development ability indirectly affects environmental performance by influencing green dual interaction dimension.
  H3b: green dual balance dimension plays a mediating role in the process of the influence of dynamic sustainable development ability on environmental performance; that is, dynamic sustainable development ability indirectly affects environmental performance by influencing green dual balance dimension.

*(3) The Mediating Role of Low-Carbon Manufacturing Practice.* Low-carbon manufacturing practice means that manufacturing enterprises develop and use new green energy to replace traditional nonrenewable energy and reduce carbon emissions. As China pays more attention to environmental protection, the pressure on manufacturing enterprises to reduce carbon emissions increases [24–26]. At the same time, more and more scholars also turn their attention to the new field of low-carbon manufacturing, and study the proposition from different angles. Some scholars have successfully transferred from the exploration of manufacturing strategy to the research of low-carbon manufacturing practice. The implementation of low-carbon manufacturing strategy may not bring immediate economic benefits to manufacturing enterprises, but the practice of low-carbon manufacturing belongs to the model of sustainable development, which is an organic development model that coordinates the overall situation, reduces resource use and waste, and reduces carbon dioxide emissions [26]. The implementation of low-carbon manufacturing practice can effectively reduce the waste of resources and environmental pollution caused by emissions, save the cost of manufacturing enterprises and the necessary investment of manufacturing enterprises to eliminate their own negative influence on the environment to a certain extent, and indirectly promote the environmental benefits and environmental performance of manufacturing enterprises [24, 25]. Under the framework of dynamic sustainable development, the concept of green development will imperceptibly affect the behavior of manufacturing enterprises, create the good atmosphere for energy conservation and emission reduction, promote manufacturing enterprises to actively implement low-carbon manufacturing practice, and then contribute to environmental performance. Huang et al. [24, 25] also put forward the view that low-carbon manufacturing strategy could bring sustainable competitive advantages and good economic benefits to manufacturing enterprises. In the framework of sustainable development, low-carbon strategic transformation is the necessary path for manufacturing enterprises to enhance environmental performance and obtain environmental benefits. Therefore, this paper puts forward the following theoretical hypothesis:

  H4: low-carbon manufacturing practice plays a mediating role in the process of the influence of dynamic sustainable development ability on environmental performance; that is, dynamic sustainable development ability indirectly affects environmental performance by influencing low-carbon manufacturing practice of manufacturing enterprises.

*(4) The Mediating Role of Green Intellectual Capital*. Green intellectual capital is a complex compound of various types of capital to enhance the growth of enterprise value [28–34]. Chen [29] conducted a systematic study on green intellectual capital, and made the hierarchical division of green intellectual capital from the perspective of structure, human resources, and capital. The relevant research results of Cohen and Levinthal showed that through the knowledge learning and experience training on environmental protection management for the internal personnel of the organization, the ability of employees is improved and the manufacturing enterprise is promoted to enhance environmental performance and environmental benefits [31]. Through *R* & *D* investment in the environmental management system and environmental protection, the dynamic sustainable development ability of manufacturing enterprises can be further improved, which is conducive to the further improvement of environmental performance [32]. By increasing the green capital of manufacturing enterprises, it has a significant positive influence on the green innovation performance of manufacturing enterprises [33]. The green intellectual capital of manufacturing enterprises provides the good environmental foundation for the dynamic transformation of sustainable development ability of manufacturing enterprises, and relevant research results also prove that intellectual capital can provide key strategic resources for the development of manufacturing enterprises [34] and improve environmental performance. At the same time, dynamic sustainable development ability can significantly enhance the ability of manufacturing enterprises to identify problems and opportunities, so as to promote manufacturing enterprises to identify key green resources and increase investment, optimize the green intellectual capital of manufacturing enterprises, and finally achieve the goal of promoting environmental performance. Under the guidance of dynamic and sustainable development of manufacturing enterprises, accumulating strategic resources, and activating and using green intellectual capital can significantly improve the environmental performance. Therefore, this paper puts forward the following theoretical hypothesis:

  H5: green intellectual capital plays a mediating role in the process of the influence of dynamic sustainable development ability on environmental performance; that is, dynamic sustainable development ability indirectly affects environmental performance by influencing green intellectual capital.

#### 2.1.3. Moderating Roles

*(1) The Moderating Role of Environmental Regulation*. Environmental regulation means that the government designs and regulates environmental standards to implement an economic intervention in order to achieve the relatively balanced state between environmental protection and economic development [34–36]. Scholars mainly study and deeply discuss the related propositions of environmental regulation from three aspects: the concept, category, and application means of environmental regulation. Environmental protection and rational utilization of green environmental resources are the fundamental purpose of environmental regulation [34–36]. The government directly or indirectly intervenes in the economic activities of manufacturing enterprises from two aspects: mandatory environmental regulation and incentive environmental regulation. Incentive environmental regulation aims to enhance the correlations among carbon reduction, pollution discharge, other behaviors, and the economic interests of manufacturing enterprises, guide manufacturing enterprises to rationally allocate resources between the management environment and business, and implement regulation mainly through subsidies, pollution discharge, and product taxes [37]. Mandatory environmental regulation means that the government directly intervenes in the enterprise activities by means of command control, including formulating various mandatory standards and policies. Many manufacturing enterprises in transition are not aware of the importance of green resources to their environmental performance, and lack the ability to identify, absorb, integrate, and allocate green resources. Through environmental regulation, the government can directly or indirectly intervene the economic activities of manufacturing enterprises, guide manufacturing enterprises to integrate and reasonably allocate green resources, promote manufacturing enterprises to better implement low-carbon manufacturing practice, encourage or force manufacturing enterprises to pay attention to environmental protection, develop green new products, increase green intellectual capital investment, and achieve green dual interaction and green dual balance, and help manufacturing enterprises improve their market competitiveness and increase their environmental benefits and environmental performance. Therefore, this paper puts forward the following theoretical hypotheses:

  H6: environmental regulation significantly positively moderates the relationships among green resource integration ability, green intellectual capital, green dual interaction dimension, green dual balance dimension, low-carbon manufacturing practice, and environmental performance; that is, the stronger the environmental regulation, the stronger the positive influence of green resource integration ability, green intellectual capital, green duality, and low-carbon manufacturing practice on environmental performance (outcome variable).
  H6a: environmental regulation significantly moderates the relationships between the mediating variable green resource integration ability and environmental performance.
  H6b: environmental regulation significantly moderates the relationships between the mediating variable green intellectual capital and environmental performance.
  H6c: environmental regulation significantly moderates the relationships between the mediating variable green duality (green dual interaction dimension and green dual balance dimension) and environmental performance.
  H6d: environmental regulation significantly moderates the relationships between the mediating variable low-carbon manufacturing practice and environmental performance.

*(2) The Moderating Role of Forward-Looking Environmental Strategy*. Ordinary environmental strategies only put emphasis on the reduction of negative influences on the environment in the process of production activities, which do not emphasize and advocate prefortification. Sharma and Vredenburg [38] classified environmental strategies, one of which was forward-looking environmental strategies. Based on the framework of sustainable development, forward-looking environmental strategy takes active measures to prevent or reduce the adverse influence on the ecological and natural environment caused by the manufacturing enterprise in the process of business activities, or quickly judges the risks and takes measures [39]. The formulation and implementation of forward-looking environmental strategies by manufacturing enterprises can create the good atmosphere for all members to participate in green management. Participating in environmental protection projects can imperceptibly deepen the awareness of energy conservation and emission reduction, promote manufacturing enterprises to enhance their ability to integrate green resources, and then enhance the improvement of environmental performance. At the same time, manufacturing enterprises can also enhance their innovation ability, develop green products and services to adapt to the development of the trend and the needs of the public, achieve green dual interaction and balance, advocate low-carbon manufacturing practice, and finally achieve the goal of improving environmental performance. In addition, many relevant research results show that the formulation and smooth implementation of forward-looking environmental strategy can enhance manufacturing organizational cohesion, organizational belonging, organizational commitment, and self-efficacy, drive the organizational citizenship behavior within the manufacturing enterprise, increase the investment of green intellectual capital, and promote the improvement of environmental performance. Based on the above three theoretical analysis results, this paper puts forward the following theoretical hypotheses:

  H7: forward-looking environmental strategy can significantly and positively moderate the positive influence of mediating variables (green resource integration ability, green intellectual capital, green duality, and low-carbon manufacturing practice) on environmental performance (outcome variable).
  H7a: forward-looking environmental strategy significantly positively moderates the relationships between green resource integration ability and environmental performance.
  H7b: forward-looking environmental strategy significantly positively moderates the relationships between green intellectual capital and environmental performance.
  H7c: forward-looking environmental strategy significantly positively moderates the relationships between green duality (green dual interaction dimension and green dual balance dimension) and environmental performance.
  H7d: forward-looking environmental strategy significantly positively moderates the relationships between low-carbon manufacturing practice and environmental performance.

#### 2.1.4. The Moderated Mediation Effects

Under the theoretical hypotheses of H2 (green resource integration ability plays a mediating role in the influence of dynamic sustainable development ability on environmental performance), H3 (green duality plays a mediating role in the influence of dynamic sustainable development ability on environmental performance), H4 (low-carbon manufacturing practice plays a mediating role in the influence of dynamic sustainable development ability on environmental performance), H5 (green intellectual capital plays a mediating role in the influence of dynamic sustainable development ability on environmental performance), H6 (environmental regulation significantly positively moderates the relationships among green resource integration ability, green intellectual capital, green duality, low-carbon manufacturing practice, and environmental performance), and H7 (forward-looking environmental strategy can significantly and positively moderate the positive influence of mediating variables (green resource integration ability, green intellectual capital, green duality, and low-carbon manufacturing practice) on environmental performance), based on the location of mediating variables and moderating variables (mediating variables are behind the moderating variables), the influence path of variables, the direction of variable influence (positive mediating effect, positive moderating effect, and positive main effect), and the intensity of variable influence (mediating variables have significant mediating effect, and moderating variables have significant moderating effects), it is further proposed that forward-looking environmental strategy and environmental regulation significantly and positively moderate the mediating roles of green resource integration ability, green intellectual capital, green duality, and low-carbon manufacturing practice. This study puts forward the following theoretical hypotheses:

  H8: antecedent variable (dynamic sustainable development ability), mediating variables (green resource integration ability, green intellectual capital, green duality, and low-carbon manufacturing practice), moderating variable (environmental regulation), and outcome variable (environmental performance) constitute the moderated mediation role model, which plays the moderated mediation effects. Moderating variable named environmental regulation significantly positively moderates the mediating variables (green resource integration ability, green intellectual capital, green duality, and low-carbon manufacturing practice) between dynamic sustainable development ability and environmental performance.
  H8a: environmental regulation significantly positively moderates the mediating role of green resource integration ability between dynamic sustainable development ability and environmental performance, which has the moderated mediation effects.
  H8b: environmental regulation significantly positively moderates the mediating role of green intellectual capital between dynamic sustainable development ability and environmental performance, which has the moderated mediation effects.
  H8c: environmental regulation significantly positively moderates the mediating role of green duality (green dual interaction dimension and green dual balance dimension) between dynamic sustainable development ability and environmental performance, which has the moderated mediation effects.
  H8d: environmental regulation significantly positively moderates the mediating role of low-carbon manufacturing practice between dynamic sustainable development ability and environmental performance, which has the moderated mediation effects.
  H9: antecedent variable (dynamic sustainable development ability), mediating variables (green resource integration ability, green intellectual capital, green duality, and low-carbon manufacturing practice), moderating variable named forward-looking environmental strategy, and outcome variable (environmental performance) constitute the moderated mediation role model to play the moderated mediation effects; the moderating variable named forward-looking environmental strategy significantly positively moderates the mediating variables (green resource integration ability, green intellectual capital, green duality, low-carbon manufacturing practice) between dynamic sustainable development ability and environmental performance.
  H9a: forward-looking environmental strategy significantly positively moderates the mediating role of green resource integration ability between dynamic sustainable development ability and environmental performance, which has the moderated mediation effects.
  H9b: forward-looking environmental strategy significantly positively moderates the mediating role of green intellectual capital between dynamic sustainable development ability and environmental performance, which has the moderated mediation effects.
  H9c: forward-looking environmental strategy significantly positively moderates the mediating role of green duality (green dual interaction dimension and green dual balance dimension) between dynamic sustainable development ability and environmental performance, which has the moderated mediation effects.
  H9d: forward-looking environmental strategy significantly positively moderates the mediating role of low-carbon manufacturing practice between dynamic sustainable development ability and environmental performance, which has the moderated mediation effects.

### 2.2. Conceptual Model Construction

According to the theoretical hypothesis of the direct relationships between dynamic sustainable development ability and environmental performance, the theoretical hypothesis of mediating role, the theoretical hypothesis of moderating role, and the theoretical hypothesis of the moderated mediation role, the conceptual model of the black-box deconstruction of dynamic sustainable development ability driving environmental performance is constructed. The conceptual model is shown in Figure 1. The conceptual model reflects and characterizes the influence mechanism of dynamic sustainable development ability on environmental performance of manufacturing enterprises.

## 3. Research Design

### 3.1. Scale Measurement

This study draws on the research results of relevant literature and sets up the scales of mediating variables and moderating variables. The existing relevant research results show that a large number of scholars have studied the contents related to dynamic sustainable development ability and environmental performance, and obtained consistent conclusions [1–43]. The reliability and validity of the scales have been widely recognized. In this paper, the evaluation index values corresponding to dynamic sustainable development ability and environmental performance scales are averaged.

Based on the study of relevant literature, the maturity scale of Rao [14] was cited to construct the scale of green resource integration ability (GICP), which acted as mediating variable. There are four measurement items in total. The specific measurement items are shown in Table 1.

On the basis of the research papers on the constituent elements of green duality, the research results of Zhou and Wu [21], Kollmann and Stockmann [22], and Xue [16] were used to measure green duality from the two dimensions of green exploration and green utilization, which are shown in Table 2 for details. Referring to and drawing on relevant research results, the concepts of green exploration and green utilization in duality are introduced into the green innovation practice [16]. Green exploration *x* and green utilization *y* are organically combined to study green duality from the balance and interaction dimensions. Referring to the existing achievements, the mathematical expression *x* × *y* reflects the interaction dimension of green exploration and green utilization [18]. The mathematical expression 1 − |*x* − *y*|/(*x*+*y*) represents the balance dimension of green exploration and green utilization [18]. GID refers to green dual interaction dimension, which is called green dual interaction for short. GBD represents the green dual balance dimension, which is called green dual balance for short.

The scale design of the mediating variable green intellectual capital was mainly based on the relevant research results of Chen [29], Cohen and Levinthal [31], Stewart [28], which was further adjusted appropriately according to the research titles, research situations, and research purposes. The specific items are shown in Table 3.

According to the existing relevant research results [23–27], the mediating variable low-carbon manufacturing practice items were screened and adjusted according to the research objects of this paper. The specific items are shown in Table 4.

Based on the relevant literature [34–37], and in combination with various environmental documents issued by the governments, the environmental regulation scale was constructed. The items are shown in Table 5.

The determination of forward-looking environmental strategy scale was mainly based on the relevant research results of Buysse and Verbeke [43], and Pan and Tian [34]. The specific measurement items are shown in Table 6.

### 3.2. Questionnaire Design, Reliability, and Validity Analyses

#### 3.2.1. Questionnaire Design and Distribution

This study consists of eight variables. The dynamic sustainable development ability of manufacturing enterprises DS is set as antecedent variable, and the environmental performance EP is set as outcome variable. Four mediating variables GICP, GIC, GD, and LCMP are selected as green resource integration ability, green intellectual capital, green duality, and low-carbon manufacturing practice, respectively, and two moderating variables ER and FES are selected as environmental regulation and forward-looking environmental strategy, respectively. In order to ensure the applicability, validity, and content validity of the scales, the scales used in this paper are mature scales that have been studied home and abroad. According to the current situations and research purposes, the scales are modified and adjusted according to the circumstances in China. In this paper, the firsthand questionnaire survey data and statistical data are obtained by means of questionnaire survey. The electronic version of the questionnaire is delivered and transferred through modern communication tools and communication technology, professional questionnaire survey websites, professional questionnaire survey institutions, network media, etc. On the basis of integrating the online distribution of the questionnaire, this study completes the questionnaire survey through the offline distribution channels (field interview, field survey, offline distribution, and post office questionnaire). The online distribution of questionnaires is mainly realized by email, online link delivery of questionnaires, relevant professional survey websites, and institutions. Offline research work is mainly completed through field interviews and field survey questionnaires. The items of the questionnaire were measured by 5-point Likert scale, and the corresponding values were 1 to 5 from small to large according to the degree of influence/effect/consent. In this study, 600 questionnaires were distributed, 531 were recovered, 62 were invalid, 469 were valid, and the effective rate was 78.17%. This study strictly controlled the common method deviation from the procedures, enhanced the readability, comprehensibility, and practicality of the questionnaire items, prevented self-report of the respondents, psychological cognitive deviation, self-concern, social approval, and other phenomena, and ensured the validity and reliability of the scale data. Harman's single-factor analysis method is used to test the common method deviation. The common method deviation test results show that the corresponding value of the maximum common factor variance interpretation rate is 26.307%, seven common factors are extracted, the characteristic roots of the seven common factors in the gravel map are higher than 1, and the maximum common factor variance interpretation rate is less than 40% of the specified value. There is no serious common method deviation in this study.

#### 3.2.2. Survey Sample and Sample Characteristics

The survey sample and empirical research sample of this paper mainly involve the representative and typical manufacturing enterprises in the eastern and central regions. In order to guarantee the validity and reliability of the scale data and ensure that the respondents' knowledge and experience can effectively reflect the real situation of manufacturing enterprises, the surveyed enterprises are manufacturing enterprises with more than 10 years and the respondents are middle and senior managers who have worked for more than 10 years.  Table 7 shows the statistical data of the survey sample and empirical research sample. The vast majority of the surveyed enterprises are large- and medium-sized manufacturing enterprises, of which enterprises with more than 500 people account for 47.34% (sample number 222), and enterprises with 301–500 people account for 18.76% (sample number 88). The surveyed enterprises are mainly private enterprises, and state-owned and state-owned holding enterprises, of which private enterprises account for 47.76% (224 samples), and state-owned and state-owned holding enterprises account for 18.12% (85 samples). In order to further ensure the validity and authenticity of the primary statistical data source, the respondents mainly focused on the middle and senior managers who are familiar with the production and operation, environmental performance, and environmental management of the manufacturing enterprise. The middle managers account for 52.88% (248 samples), and the senior managers account for 47.12% (221 samples). The educational background of the respondents mainly concentrates in undergraduate and above, accounting for 73.99%.

#### 3.2.3. Scale Reliability Test

This study adopts two indexes CITC (Churchill's standard, deletion of invalid indicators, and operating guidelines) and Cronbach's coefficient (Nunnally's standard) of the research sample to measure the reliability level of the scale [49–51]. The reliability analysis results of the overall and local scales are shown in Table 8. The Cronbach coefficient values are between 0.838 and 0.921, which are higher than 0.8. The CITC values of scale are between 0.674 and 0.830, which are higher than 0.50. The Cronbach coefficient after deleting the project does not highlight the obvious growth trend and significant change trend. Table 8 shows that the overall and local scales have good reliability.

#### 3.2.4. Scale Validity Test

The overall and local scale validity test results are shown in Table 9. The KMO values corresponding to the scale variables of green resource integration ability, green intellectual capital, green duality, low-carbon manufacturing practice, environmental regulation, and forward-looking environmental strategy are between 0.711 and 0.938, which are higher than 0.7. The combination reliability values of CFA statistics corresponding to green resource integration ability, green intellectual capital, green duality, low-carbon manufacturing practice, environmental regulation, and forward-looking environmental strategy are between 0.8390 and 0.9353, which are all higher than 0.6. The AVE values of CFA statistics corresponding to green resource integration ability, green intellectual capital, green duality, low-carbon manufacturing practice, environmental regulation, and forward-looking environmental strategy are between 0.6304 and 0.7850, which are all higher than 0.5. And the load values of the standardization factor in the CFA scenario are between 0.732 and 0.911, which are higher than 0.6. The statistical results of Table 9 show that the scale has good validity.

## 4. Hypothesis Test of Theoretical Hypothesis

### 4.1. Main Effect and Mediating Effect Test Process and Results

The nonparametric percentile bootstrap method based on deviation correction is a nonparametric statistical method based on automatic self-help sampling, putting-back sampling, and resampling of the initial sample to estimate the total sample population. It is a reasoning method to simulate the frequency theory, and evaluate and improve the accuracy of statistical analysis and inference. The research system of the method has been greatly developed in economic and management subject fields and areas, which is often used to solve the complex problems without a theoretical basis; it is not limited to the sample size and whether the sample data conform to the normal distribution. The more the repeated sampling times are and the closer the obtained data to the original data are, the better the research results will be. The method has competence and explanatory power in verifying the main effect, the mediating effects, the moderating effects, and the moderated mediation effects, which also shows high applicability, feasibility, rationality, and effectiveness in clarifying and elaborating the influence mechanism, function mechanism, and influence paths. The nonparametric percentile bootstrap method based on deviation correction is operable, accurate, and robust in deconstructing the driving black-box and the operational black-box among variables. In this study, the nonparametric percentile bootstrap method based on deviation correction is used to empirically test the main effect and mediating effect of the relevant theoretical hypothesis in the conceptual model of the black-box of environmental performance driven by dynamic sustainable development ability (the conceptual model of the influence mechanism of dynamic sustainable development ability on environmental performance of manufacturing enterprises) (Figure 1). The test is conducted according to the main effect and mediating effect test proposed by Wen et al. [44, 45]. The following equations (1)–(3) describe the causal relationships between variables in the analysis of the main effect and mediating effect test:

(1) $$\begin{array}{c} Y=CX+e_{1}, \end{array}$$

(2) $$\begin{array}{c} M=AX+e_{2}, \end{array}$$

(3) $$\begin{array}{c} Y=C^{\prime }X+BM+e_{3}. \end{array}$$

In equation (1), *C* is the total effect of an antecedent variable *X* on outcome variable *Y*. In equation (2), *A* is the effect of an antecedent variable on mediating variable *M*. In equation (3), *B* is the effect of the mediating variable on outcome variable, and *C*′ is the effect of an antecedent variable on outcome variable after the mediating variable is introduced.

We strictly follow the mediating effect test process proposed by Wen et al. [44, 45]. Firstly, we test whether the regression coefficient *C* of the influence of antecedent variable dynamic sustainable development ability on environmental performance is significant. Secondly, we judge whether the regression coefficient *A* of antecedent variable dynamic sustainable development ability on the mediating variables and the regression coefficient *B* of the mediating variables on environmental performance are significant. Finally, after adding to mediating variables, according to the significance of regression coefficient *C*′ of antecedent variable dynamic sustainable development ability on the influence of environmental performance and the comparison results of the values between *C* and *C*′, we judge whether the mediating variables play mediating roles in the relationships between dynamic sustainable development ability and environmental performance.

The bootstrapping calculation results in Table 10 show that Model 6 shows the regression results of the influence of dynamic sustainable development ability on environmental performance of manufacturing enterprises. After controlling the control variables of the nature and size of manufacturing enterprises, dynamic sustainable development ability of manufacturing enterprises has a significant positive influence on environmental performance (*C* = 0.5511, *P* < 0.001). The hypothesis H1 has been empirically verified.

According to the three-step test and analysis process of mediating effect, we empirically test and analyze mediating variables. Firstly, the regression coefficient significances of the influences of antecedent variable dynamic sustainable development ability on the mediating variables (green resource integration ability, green intellectual capital, green duality (green dual interaction and green dual balance), and low-carbon manufacturing practice) are tested. The data in Table 10 show that the bootstrapping calculation results of Model 1, Model 2, Model 3, Model 4, and Model 5 show that the regression coefficients A of dynamic sustainable development ability on the mediating variables named green resource integration ability, green intellectual capital, green dual interaction, green dual balance, and low-carbon manufacturing practice are 0.3633, 0.3855, 1.93029, 0.0416, and 0.3002, respectively, and the *P* values are less than 0.001, indicating that dynamic sustainable development ability of the manufacturing enterprise can play significant positive roles in promoting green resource integration ability, green intellectual capital, green dual interaction, green dual balance, and low-carbon manufacturing practice.

Secondly, this study tests the significance of the influence of mediating variables on environmental performance. Table 10 shows that the bootstrapping calculation results of Model 6, Model 7, Model 8, Model 9, Model 10, and Model 11 show that the regression coefficients B of the influence of mediating variables named green resource integration ability, green intellectual capital, green dual interaction, green dual balance, and low-carbon manufacturing practice on environmental performance are 0.2549, 0.277, 0.0466, 1.7735, and 0.2139, respectively, and the *P* values are less than 0.001, indicating that green resource integration ability, green intellectual capital, green dual interaction, green dual balance, and low-carbon manufacturing practice have significant positive influences on environmental performance.

Finally, based on the significant direct effects of green resource integration ability, green intellectual capital, green dual interaction, green dual balance, and low-carbon manufacturing practice on environmental performance, the bootstrapping results of Model 6, Model 7, Model 8, Model 9, Model 10, and Model 11 show that after the participation of mediating variables, the direct effect of dynamic sustainable development ability of manufacturing enterprises on environmental performance *C*′ is significant (although compared with Model 6, the value decreases slightly, but still remains significant). *AB* and *C*′ maintain the same sign relationships, which further shows that green resource integration ability, green intellectual capital, green dual interaction, green dual balance, and low-carbon manufacturing practice play partially mediating effects between dynamic sustainable development ability of manufacturing enterprises and environmental performance. It is assumed that H2, H3a, H3b, H4, and H5 are demonstrated.

### 4.2. Moderating Effect Test Process and Results

According to formulas and equations (4)–(7), this study adopts the nonparametric percentile bootstrap method based on deviation correction to empirically test the moderating effect of the relevant theoretical hypothesis in the conceptual model (conceptual model of the influence mechanism of dynamic sustainable development ability on environmental performance of manufacturing enterprises) of the black-box of environmental performance driven by dynamic sustainable development ability (Figure 1). The empirical test on the moderating effect is conducted by referring to the moderating effect test process proposed by Wen et al. [44, 45]. We set outcome variable as *Y*, and carry out the standardized bootstrapping regression coefficient test (formula (5)) of the interaction term between the antecedent variable *X* and the moderating variable *U*. If the bootstrapping regression coefficient is significant, and the goodness of fit estimated by the regression model of equation (5) is higher than that estimated by the regression model of equation (4), the moderating effect is significant. On the contrary, the moderating effect is not significant.

(4) $$\begin{array}{c} Y=C_{0}^{\prime }+C_{1}^{\prime \prime }X+C_{2}^{\prime \prime }U+e_{4}, \end{array}$$

(5) $$\begin{array}{c} Y=C_{0}+C_{1}X+C_{2}U+C_{3}UX+e_{5}, \end{array}$$

(6) $$\begin{array}{c} W=A_{0}+A_{1}X+e_{6}, \end{array}$$

(7) $$\begin{array}{c} Y=C_{0}^{\prime }+C_{1}^{\prime }X+C_{2}^{\prime }U+C_{3}^{\prime }UX+B_{1}W+B_{2}UW+e_{7}. \end{array}$$

According to the moderating effect test process proposed by Wen et al., combined with the research objects of this paper, we test whether the moderating effects of moderating variables on the relationships between mediating variables and outcome variable are significant. According to the results of bootstrapping operation in Table 11, the regression coefficient of the interaction term between the mediating variable GICP and the moderating variable ER is 0.1489, the *P* value is less than 0.001, and the confidence interval is [0.1004, 0.2489], excluding 0, indicating that the interaction term has a significant influence. After introducing the interaction term, the overall *R*^2^-chng of the model is 0.0212, *P*=0.0001 < 0.001, indicating that the moderating effect of the moderating variable ER is significant, and ER significantly moderates the relationships between GICP and *Y*. The hypothesis H6a is verified. The regression coefficient of the interaction term between the mediating variable GICP and the moderating variable FES is 0.0633, the *P* value is greater than 0.1, and the confidence interval is [−0.0104, 0.1370], including 0. After introducing the interaction term, the overall *R*^2^-chng of the model is 0.0037, *P*=0.0923, which is close to 0.1 (not significant), indicating that the moderating effect of the moderating variable FES is not significant, and the hypothesis H7a is not supported.

According to the moderating effect test process proposed by Wen et al., combined with the research objects of this paper, we test whether the moderating effects of moderating variables on the relationships between mediating variables and outcome variable are significant. According to the bootstrapping regression results in Table 12, the regression coefficient of the interaction term between the mediating variable GIC and the moderating variable ER is 0.1920, the *P* value is less than 0.001, and the confidence interval is [0.1222, 0.2619], excluding 0, indicating that the interaction term has a significant influence. After introducing the interaction term between GIC and ER, the overall *R*^2^-chng of the model is 0.0361, *P*=0.0000 < 0.001, indicating that the moderating effect of the moderating variable ER is significant; that is, ER significantly moderates the relationships between GIC and *Y*, and the hypothesis H6b is verified. The regression coefficient of the interaction term between the mediating variable GIC and the moderating variable FES is 0.0433, the *P* value is greater than 0.1, and the confidence interval is [−0.0305, 0.1170], including 0. After introducing the interaction term between GIC and FES, the overall *R*^2^-chng of the model is 0.0017, *P*=0.2499 > 0.1 (not significant), indicating that the moderating effect of the moderating variable FES is not significant, and the hypothesis H7b is not supported.

According to the moderating effect test process proposed by Wen et al., combined with the research objects of this paper, we test whether the moderating effects of moderating variables on the relationships between mediating variables and outcome variable are significant. According to the bootstrapping regression results in Table 13, the regression coefficient of the interaction term between the mediating variable GID and the moderating variable ER is 0.1869, the *P* value is less than 0.001, and the confidence interval is [0.1181, 0.2556], excluding 0, which indicates that the interaction term has a significant influence. After introducing the interaction term between GID and ER, the overall *R*^2^-chng of the model is 0.0346, *P*=0.0000 < 0.001 (significant), indicating that the moderating effect of the moderating variable ER is significant; that is, ER significantly moderates the relationships between GID and *Y*, and the hypothesis H6c is verified. The regression coefficient of the interaction term between the mediating variable GID and the moderating variable FES is 0.0005, the *P* value is greater than 0.1, and the confidence interval is [−0.0708, 0.0718], including 0. After introducing the interaction term between GID and FES, the overall *R*^2^-chng of the model is 0.000, *P*=0.9894 > 0.1 (not significant), and the moderating effect of the moderating variable FES is not significant. The hypothesis H7c is not supported.

According to the moderating effect test process proposed by Wen et al., combined with the research objects of this paper, we test whether the moderating effects of moderating variables on the relationships between mediating variables and outcome variable are significant. According to the bootstrapping regression results in Table 14, the regression coefficient of the interaction term between the mediating variable GBD and the moderating variable ER is 0.1970, the *P* value is less than 0.001, and the confidence interval is [0.1245, 0.2695], excluding 0, indicating that the interaction term has a significant influence. After introducing the interactive terms GBD and ER, the overall *R*^2^-chng of the model is 0.0339, *P*=0.0000 < 0.001 (significant), indicating that the moderating effect of the moderating variable ER is significant; that is, ER significantly moderates the relationships between GBD and *Y*, and the hypothesis H6c is verified. The regression coefficient of the interaction term between the mediating variable GBD and the moderating variable FES is 0.00263, the *P* value is greater than 0.1 (not significant), and the confidence interval is [−0.0625, 0.0766], including 0. After introducing the interaction term between GBD and FES, the overall *R*^2^-chng of the model is 0.0007, and *P*=0.076 is close to 0.1 (the change is not significant). The moderating effect of the moderating variable FES is not significant, and the hypothesis H7c is not supported.

According to the moderating effect test process proposed by Wen et al., combined with the research objects of this paper, we test whether the moderating effects of moderating variables on the relationships between mediating variables and outcome variable are significant. According to the bootstrapping regression results in Table 15, the regression coefficient of the interaction term between the mediating variable LCMP and the moderating variable ER is 0.2044, the *P* value is less than 0.001, and the confidence interval is [0.1329, 0.2759], excluding 0, indicating that the interaction term has a significant influence. After introducing the interaction term between LCMP and ER, the overall *R*^2^-chng of the model is 0.0396 and *P*=0.0000 < 0.001 (significant), indicating that the moderating effect of the moderating variable ER is significant; that is, ER significantly moderates the relationships between LCMP and *Y*, and the hypothesis H6d is verified. The regression coefficient of the interaction term between the mediating variable LCMP and the moderating variable FES is 0.0690, the *P* value is greater than 0.1, and the confidence interval is [−0.0073, 0.1454], including 0. After introducing the interaction term between GIC and FES, the overall *R*^2^-chng of the model is 0.0042, *P*=0.4566 > 0.1 (not significant), and the moderating effect of the moderating variable FES is not significant. The hypothesis H7d is not supported.

### 4.3. The Process and Results of the Moderated Mediation Effect Test

According to formulas and equations (4)–(7), this study adopts the nonparametric percentile bootstrap method based on deviation correction to empirically test the moderated mediation effect by the relevant theoretical hypothesis in the conceptual model of the black-box of environmental performance of manufacturing enterprises driven by dynamic sustainable development ability (the conceptual model of the influence mechanism of dynamic sustainable development ability on environmental performance of manufacturing enterprises) (Figure 1). For the mediation model test in the second half of the moderated period, we will empirically test the moderated effect by referring to the test process proposed by Wen et al. [44, 45]. We use the regression model with interactive product term to perform bootstrapping operation: firstly, we check whether the regression coefficients *A*1 of the influences of an antecedent variable on the mediating variables and the regression coefficients *B*2 of the interactions between the mediating variables and the moderating variables are significant and whether the confidence interval contains 0. If the regression coefficients are significant and the confidence interval does not contain 0, it indicates that the mediating effect is moderated by the moderating variable. And further, this study reports the influence on the mean value of the moderating variable, the mediating effect ranges corresponding to the differences between positive and negative standard deviations, and its groups. The model only moderates the second half of the mediating effect; it is also necessary to report the index value and its confidence interval corresponding to the moderating variable. The index indicates the influence of the moderating variable on the whole mediation path. If the index value is positive and the confidence interval does not contain 0, it indicates that the moderated mediation effect is significant. In addition, if the coefficient of the interaction term is not significant, and the confidence interval corresponding to the regression coefficient of the interaction product term contains 0, it is necessary to continue to test the confidence interval of the differences between the maximum value and minimum value of the mediating effect. If the above confidence interval does not contain 0, the mediating effect is moderated by the moderating role. On the contrary, the mediating effect is not moderated by the moderating role.

According to the moderating effect test, the hypothesis H7 is not supported. Therefore, the hypothesis H9 will not be tested.

DS, GICP, ER, and EP constitute the moderated mediation effect model, and the moderated mediation effect test results are shown in Table 16. According to the moderated mediation effect test process, the regression coefficient of DS on GICP is 0.3633, and *P* value is less than 0.001, which is significant. The coefficient of interaction term between GICP and ER is further tested. According to Table 11, the regression coefficient of interaction term is 0.1489, the *P* value is less than 0.001, and the confidence interval is [0.1004, 0.2489], excluding 0. As shown in Table 16, as for the indirect effect, after introducing the moderating variable ER, the confidence intervals of DS ⟶ GICP ⟶ EP model in which GICP is moderated by ER (−1, 0, 1) are [−0.0268, 0.0642], [0.0449, 0.123], and [0.0506, 0.2021], respectively, the differences between groups are 0.1201, and the confidence interval is [0.0441, 0.1822], excluding 0, indicating that the stronger the moderating effect of ER is, the stronger the mediating effect of the mediating variable GICP is; that is, the mediating effect of GICP is positively moderated by ER. At the same time, the index of moderated mediation value of the moderating variable ER is 0.0601, and the confidence interval is [0.0253, 0.1006], excluding 0; ER produces a significant moderated mediation effect, which confirms that ER plays a moderating role in the mediated effect of GICP, and the hypothesis H8a is verified.

DS, GIC, ER, and EP constitute the moderated mediation effect model, and the moderated mediation effect test results are shown in Table 17. According to the moderated mediation effect test process, the regression coefficient of DS on GIC is 0.3855, and *P* value is less than 0.001, which is significant. The regression coefficient of interaction term between GIC and ER is further tested. According to Table 12, the coefficient of interaction term is 0.1920, *P* value is less than 0.001 (significant), and the confidence interval is [0.1222, 0.2619], excluding 0. As shown in Table 17, as for the indirect effect, after introducing the moderating variable ER, the confidence intervals of DS ⟶ GIC ⟶ EP model whose GIC is moderated by ER (−1, 0, 1) are [−0.0422, 0.0599], [0.0560, 0.1449], and [0.1259, 0.2589], respectively, the differences between groups are 0.1776, and the confidence interval is [0.1027, 0.2568], excluding 0, indicating that the stronger the moderating effect of ER, the stronger the mediating effect of the mediating variable GIC; that is, the mediating effect of GIC is positively moderated by ER. At the same time, the index of moderated mediation value of the moderating variable ER is 0.0888, and the confidence interval is [0.0514, 0.1284], excluding 0; ER produces a significant moderated mediation effect, which confirms that ER plays a moderating role in the mediated effect of GIC, and the hypothesis H8b is verified.

DS, GID, ER, and EP constitute the moderated mediation effect model. The moderated mediation effect results are shown in Table 18. According to the moderated mediation effect test process, the regression coefficient of DS on GID is 1.93029, and the *P* value is less than 0.001 (significant). Further, we test the regression coefficient of the interaction term between GID and ER. According to Table 13, the interaction term coefficient is 0.1869, the *P* value is less than 0.001 (significant), and the confidence interval is [0.1181, 0.2556], excluding 0. As shown in Table 18, as for the indirect effect, after the introduction of moderating variable ER, the confidence intervals of DS ⟶ GID ⟶ EP model whose GID is moderated by ER (−1, 0, 1) are [−0.0407, 0.0531], [0.0521, 0.1188], and [0.1161, 0.2142] respectively, the differences between groups are 0.1558, and the confidence interval is [0.0901, 0.2287], excluding 0, indicating that the stronger the moderating effect of ER, the stronger the mediating effect of the mediating variable GID; that is, the mediating effect of GID is positively moderated by ER. At the same time, the index of moderated mediation value of the moderating variable ER is 0.0779, and the confidence interval is [0.0451, 0.1144], excluding 0; ER produces a significant moderated mediation effect, which confirms that ER plays a moderating role in the mediated effect of GID, and the hypothesis H8c is verified.

DS, GBD, ER, and EP constitute the moderated mediation effect model, and the moderated mediation effect test results are shown in Table 19. According to the moderated mediation effect test process, the regression coefficient of DS on GBD is 0.0416, and the *P* value is less than 0.001 (significant). Further, we test the regression coefficient of the interaction term between GBD and ER. According to Table 14, the interaction term coefficient is 0.1970, the *P* value is less than 0.001 (significant), and the confidence interval is [0.1245, 0.2695], excluding 0. As shown in Table 19, as for the indirect effect, after introducing the moderating variable ER, the confidence intervals of DS ⟶ GBD ⟶ EP model in which GBD is moderated by ER (−1, 0, 1) are [−0.0250, 0.0540], [0.0501, 0.1231], and [0.0999, 0.2135] respectively, the differences between groups are 0.1388, and the confidence interval is [0.0788, 0.2081], excluding 0, indicating that the stronger the moderating effect of ER, the stronger the mediating effect of the mediating variable GBD; that is, the mediating effect of GBD is positively moderated by ER. At the same time, the index of moderated mediation value of the moderating variable ER is 0.0694, and the confidence interval is [0.0394, 0.1040], excluding 0; the moderated mediation effect of ER is significant, which confirms that ER plays a moderating role in the mediated effect of GBD, and the hypothesis H8c is verified.

DS, LCMP, ER, and EP constitute the moderated mediation effect model, and the moderated mediation effect test results are shown in Table 20. According to the moderated mediation effect test process, the regression coefficient of DS on LCMP is 0.3002, and the *P* value is less than 0.001 (significant). Further, we test the regression coefficient of the interaction term between LCMP and ER. It can be seen from Table 15 that the interaction term coefficient is 0.2044, the *P* value is less than 0.001, which is significant, and the confidence interval is [0.1329, 0.2759], excluding 0. As shown in Table 20, as for the indirect effect, after introducing the moderating variable ER, the confidence intervals of DS ⟶ LCMP ⟶ EP model in which LCMP is moderated by ER (−1, 0, 1) are [−0.0634, 0.0185], [0.0203, 0.0876], and [0.0767, 0.1817] respectively, the differences between groups are 0.1474, and the confidence interval is [0.0839, 0.2180], excluding 0, indicating that the stronger the moderating effect of ER is, and the stronger the mediating effect of the mediating variable LCMP is, the mediating effect of LCMP is positively moderated by ER. At the same time, the index of moderated mediation value of the moderating variable ER is 0.0737, and the confidence interval is [0.0419, 0.1090], excluding 0. ER produces a significant moderated mediation effect, which confirms that ER plays a moderating role in the mediated effect of LCMP. The hypothesis H8d is verified.

## 5. Research Conclusion and Enlightenment

### 5.1. Research Conclusion

This paper takes 469 representative and typical manufacturing enterprises in the eastern and central regions as the empirical analysis objects, adopts the nonparametric percentile bootstrap method based on deviation correction to empirically complete the research goals of revealing the influence mechanism of dynamic sustainable development ability on environmental performance of manufacturing enterprises and empirically deconstructing the black-box of dynamic sustainable development ability driving environmental performance of manufacturing enterprises, and further empirically discusses the mediating roles of green resource integration ability, green duality, low-carbon manufacturing practice, and green intellectual capital, as well as the moderating roles of environmental regulation and forward-looking environmental strategy. The main empirical analysis conclusions are as follows: (1) main effect—dynamic sustainable development ability has a significant positive influence on environmental performance of manufacturing enterprises; (2) mediating effects—dynamic sustainable development ability affects environmental performance of manufacturing enterprises through green resource integration ability, which is integrated into the mediating mechanism model of dynamic sustainable development ability ⟶ green resource integration ability ⟶ environmental performance; that is, dynamic sustainable development ability indirectly affects environmental performance by affecting green resource integration ability. Dynamic sustainable development ability has influence on environmental performance through green duality, which is integrated into the mediating mechanism model of dynamic sustainable development ability ⟶ green duality ⟶ environmental performance; that is, dynamic sustainable development ability has indirect influence on environmental performance through green duality. Dynamic sustainable development ability has positive influence on environmental performance through low-carbon manufacturing practice, which is integrated into the mediating mechanism model of dynamic sustainable development ability ⟶ low-carbon manufacturing practice ⟶ environmental performance; that is, dynamic sustainable development ability has an indirect influence on environmental performance through influencing low-carbon manufacturing practice. Dynamic sustainable development ability has an influence on environmental performance through green intellectual capital, which is integrated into the mediating mechanism model of dynamic sustainable development ability ⟶ green intellectual capital ⟶ environmental performance; that is, dynamic sustainable development ability has an indirect influence on environmental performance through green intellectual capital; (3) moderating effects—environmental regulation significantly positively moderates the relationships among green resource integration ability, green duality, low-carbon manufacturing practice, green intellectual capital, and environmental performance; and (4) moderated mediation effects—environmental regulation, as the boundary condition, plays the buffer function. Environmental regulation significantly positively moderates the mediating mechanism and mediating transmission paths of green resource integration ability, green duality, low-carbon manufacturing practice, and green intellectual capital of the relationships between dynamic sustainable development ability and environmental performance of manufacturing enterprises; namely, environmental regulation significantly positively moderates the mediating function of green resource integration ability of the relationships between dynamic sustainable development ability and environmental performance of manufacturing enterprises; environmental regulation significantly positively moderates the mediating function of green duality of the relationships between dynamic sustainable development ability and environmental performance of manufacturing enterprises; environmental regulation significantly positively moderates the mediating function of low-carbon manufacturing practice of the relationships between dynamic sustainable development ability and environmental performance of manufacturing enterprises; and environmental regulation significantly positively moderates the mediating function of green intellectual capital of the relationships between dynamic sustainable development ability and environmental performance of manufacturing enterprises. The stronger the environmental regulation is, the more significant the mediating function and effects of green resource integration ability, green duality, low-carbon manufacturing practice, and green intellectual capital of the relationships between dynamic sustainable development ability and environmental performance of manufacturing enterprises are.

The advantages of this paper lie in adopting the nonparametric percentile bootstrap method based on deviation correction to empirically reveal the influence mechanism of dynamic sustainable development ability on environmental performance of manufacturing enterprises, empirically deconstruct the black-box of dynamic sustainable development ability driving environmental performance of manufacturing enterprises, and empirically discuss the mediating roles of green resource integration ability, green duality, low-carbon manufacturing practice, and green intellectual capital, as well as the moderating roles of environmental regulation and forward-looking environmental strategy. Further, the main effect, the mediating effects, the moderating effects, and the moderated mediation effects are carried out.

### 5.2. Theoretical Contribution

Firstly, this study enriches and deepens the achievements in the research fields of dynamic sustainable development ability and environmental performance, effectively echoes the research themes of Maconachie and Conteh [49], sets environmental regulation and forward-looking environmental strategy as situational variables and moderating variables (boundary conditions), and defines green resource integration ability, green duality, green intellectual capital, and low-carbon manufacturing practice as mediating variables, puts emphasis on the black-box of dynamic sustainable development ability driving environmental performance of manufacturing enterprises, and empirically reveals the influence mechanism and conducting paths of dynamic sustainable development ability on environmental performance of manufacturing enterprises. Secondly, combining with the practice of manufacturing enterprises, this study extends the sustainable development ability to dynamic sustainable development ability. In view of the previous research results focusing on the direct influence of sustainable development ability of manufacturing enterprise on environmental performance, this study deeply discusses the mediating function mechanism among green resource integration ability, green duality, green intellectual capital, and low-carbon manufacturing practice, and enriches the research results on how dynamic sustainable development ability of manufacturing enterprise indirectly affects environmental performance. Finally, the research results on situational variables and boundary conditions of environmental regulation and forward-looking environmental strategy have important enlightenment significance for manufacturing enterprises to obtain environmental performance. Environmental regulation can effectively eliminate the negative environmental behavior of manufacturing enterprises, promote manufacturing enterprises to carry out green management, construct and improve dynamic sustainable development ability, and obtain environmental performance. However, in the empirical analysis, the moderating effect of forward-looking environmental strategy has not been empirically verified; it may be that manufacturing enterprises do not pay enough attention to the relevant issues of environmental strategic management from the perspective of dynamic development and future evolution, which also provides experience for the future environmental management of manufacturing enterprises.

### 5.3. Research Enlightenment

The main practical implications of this study are as follows: (1) Manufacturing enterprises should pay attention to activate green resource integration ability, identify the key green resources, and improve environmental performance. (2) It is necessary to put emphasis on the accumulation of green intellectual capital, stimulate green human capital, strengthen green structural capital and green relational capital, promote the long-term coordinated and coupled development among the three types of green intellectual capital, and give full play to the value of enterprise green intellectual capital. (3) If manufacturing enterprises want to achieve bilateral transformation and high-quality development, they should take the relationships between human needs and environmental supportability into account, and they must pay attention to the implementation of green duality practice. Based on the natural resource-based management theory, manufacturing enterprises should promote green exploration and green utilization activities and behaviors as a whole. (4) The implementation of low-carbon manufacturing practice is one of the necessary conditions for manufacturing enterprises to achieve bilateral transformation. Manufacturing enterprises should regularly conduct low-carbon production knowledge training for managers and employees to imperceptibly optimize the low-carbon thinking mode and low-carbon behavior of employees in manufacturing enterprises. (5) Through active environmental management behaviors and activities, manufacturing enterprises can strive for the support of environmental regulation and imperceptibly improve their environmental performance.

### 5.4. Research Limitations and Prospects

This research may ignore the other mediating variables and moderating variables, which may not fully reveal the influence mechanism of dynamic sustainable development ability on environmental performance of manufacturing enterprises and explore the black-box of dynamic sustainable development ability driving environmental performance of manufacturing enterprises. This research uses cross-sectional data to carry out empirical analysis of the black-box of dynamic sustainable development ability driving environmental performance of manufacturing enterprises, which may not comprehensively reveal the causal relationships among variables. In the future, we will introduce more reasonable mediating variables and moderating variables to improve and enrich the conceptual model and theoretical framework of deconstructing the black-box of dynamic sustainable development ability driving environmental performance of manufacturing enterprises, and we will also use longitudinal dynamic tracking data to carry out empirical analysis of the influence mechanism of dynamic sustainable development ability on environmental performance of manufacturing enterprises and deeply deconstruct the black-box of dynamic sustainable development ability driving environmental performance of manufacturing enterprises.

## Figures and Tables

**Figure 1:** Conceptual model.

**Table 1:** Green resource integration ability scale.

Variable name	Item	Reference
Green resource integration ability (GICP)	Identifying ability of enterprise green resources (GICP1)	Rao [14]
	Ability to absorb enterprise green resources (GICP2)	
	Enterprise green resource allocation ability (GICP3)	
	Enterprise green resource integration ability (GICP4)	

**Table 2:** Green duality scale.

Variable name		Item	Reference
Green duality (GD)	Green exploration (GEL)	Respond to green demand of customers for exceeding existing products/services (GEL1)	Zhou and Wu [21], Kollmann and Stockmann [22], Xue [16]
		Willingness to learn advanced green process technologies in the field (GEL2)	
		Develop green and environmentally friendly products/services (GEL3)	
	Green utilization (GEP)	Utilization of existing green schemes (GEP1)	
		The knowledge reserve of green technology is constantly updated and expanded (GEP2)	
		Willingness to improve the efficiency of developing green services and products (GEP3)	

**Table 3:** Green intellectual capital scale.

Variable name	Item	Reference
Green intellectual capital (GIC)	Productivity and contribution of employees in environmental protection (GIC1)	Cohen and Levinthal [29], Stewart [28], Sun [27], Pan [51]
	Each department is willing to compromise for the same environmental protection goal (GIC2)	
	Managers provide comprehensive support for employees to achieve environmental protection objectives (GIC3)	
	The perfection of enterprise environmental management system (GIC4)	
	Income from environmental protection (GIC5)	
	R & D investment of enterprises in environmental protection (GIC6)	
	Ability to research green products of enterprises (GIC7)	
	Customers are satisfied with relevant environmental protection practice of enterprise (GIC8)	

**Table 4:** Low-carbon manufacturing practice scale.

Variable name	Item	Reference
Low-carbon manufacturing practice (LCMP)	Middle and senior managers support for carbon emission reduction actions (LCMP1)	Cao [23], Hang et al. [24, 25], Cheng and Sun [26], Sun [27]
	Establishment of carbon emission reduction institutions and full-time personnel (LCMP2)	
	Conduct relevant knowledge and skills training (LCMP3)	
	Total quality management plan (LCMP4)	
	Implement collaborative waste disposal with cooperative enterprises (LCMP5)	
	Implementation degree of technical requirements for environmental labeling products (LCMP6)	
	The perfection of clean development mechanism (CDM) (LCMP7)	
	Implementation degree of environmental management system certification (LCMP8)	

**Table 5:** Environmental regulation scale.

Variable name	Item	Reference
Environmental regulation (ER)	Influence of carbon emission reduction tax reduction policy on enterprises (ER1)	Pan and Tian [34], Chen [35], Feng [36], Zhang [37]
	Influence of emission tax reduction policy on enterprises (ER2)	
	Influence of special scientific research funds for technological transformation projects on enterprises (ER3)	
	Influence of carbon emission reduction laws, decrees, and regulations on enterprises (ER4)	

**Table 6:** Forward-looking environmental strategy scale.

Variable name	Item	Reference
Forward-looking environmental strategy (FES)	Conduct environmental review on participating in environmental protection projects of government or nongovernmental organizations (FES1)	Buysse and Verbeke [43], Pan and Tian [34]
	Purchase industrial ecology protection standard manual (FES2)	
	Internal and external disclosure of environmental information (FES3)	

**Table 7:** Information of surveyed enterprises and respondents.

Information of surveyed enterprises		Number of samples	Percentage (%)

Enterprise size	≤100 persons	69	14.71
	101–300 persons	90	19.19
	301–500 persons	88	18.76
	501–1000 persons	126	26.87
	>1000 persons	96	20.47

Enterprise nature	State-owned and state-owned holding enterprises	85	18.12
	Private enterprises	224	47.76
	Foreign joint enterprises	66	14.07
	Foreign-owned enterprises	20	4.26
	Other types of enterprises	74	15.78

Respondent information		Number of samples	Percentage (%)

Post	Senior managers	221	47.12
	Middle managers	248	52.88

Education	Junior college degree	122	26.01
	Bachelor's degree	267	56.93
	Master's degree	80	17.06

**Table 8:** Internal consistency test of various scales.

Variables		Items	CITC	Cronbach's coefficient
Green resource integration ability (GICP)		GICP1	0.684	0.866
		GICP2	0.764	
		GICP3	0.719	
		GICP4	0.703	

Green intellectual capital (GIC)		GIC1	0.703	0.921
		GIC2	0.707	
		GIC3	0.731	
		GIC4	0.830	
		GIC5	0.739	
		GIC6	0.723	
		GIC7	0.732	
		GIC8	0.713	

Green duality (GD)	Green exploration (GEL)	GEL1	0.771	0.884
		GEL2	0.792	
		GEL3	0.762	
	Green utilization	GEP1	0.742	
	(GEP)	GEP2	0.769	
		GEP3	0.754	

Low-carbon manufacturing practice (LCMP)		LCMP1	0.674	0.916
		LCMP2	0.761	
		LCMP3	0.716	
		LCMP4	0.704	
		LCMP5	0.725	
		LCMP6	0.758	
		LCMP7	0.741	
		LCMP8	0.706	

Environmental regulation (ER)		ER1	0.705	0.858
		ER2	0.740	
		ER3	0.677	
		ER4	0.691	

Forward-looking environmental strategy (FES)		FES1	0.676	0.838
		FES2	0.753	
		FES3	0.678	

**Table 9:** Test results of scale validity.

Variables		KMO	Composite reliability (CR)	AVE	Factor loading
Green resource integration ability		0.829	0.9089	0.7140	0.822–0.876
Green intellectual capital		0.931	0.9353	0.6442	0.775–0.879
Green duality	Green exploration	0.741	0.8390	0.6430	0.895–0.911
	Green utilization	0.841	0.9160	0.7850	0.885–0.901
Low-carbon manufacturing practice		0.938	0.9317	0.6304	0.750–0.824
Environmental regulation		0.827	0.9039	0.7017	0.819–0.839
Forward-looking environmental strategy		0.711	0.9029	0.7562	0.732–0.808

**Table 10:** Hierarchical regression results.

Variables	Variables	GICP	GIC	GID	GBD	LCMP	EP					
		Model 1	Model 2	Model 3	Model 4	Model 5	Model 6	Model 7	Model 8	Model 9	Model 10	Model 11
Control variables	Enterprise nature	0.1662^*∗∗∗*^	0.1215^*∗∗∗*^	−0.1347	−0.0043	0.0995^*∗∗∗*^	0.0228	0.065^*∗*^	0.0108	−0.0166	−0.0152	−0.0016
	Enterprise size	−0.389	0.036	0.426^*∗*^	0.0229^*∗∗∗*^	−0.0021	0.0529	0.0628	0.4249	0.0323	0.0123	0.0533

Antecedent variable	DS	0.3633^*∗∗∗*^	0.3855^*∗∗∗*^	1.93029^*∗∗∗*^	0.0416 ^*∗∗∗*^	0.3002^*∗∗∗*^	0.5511^*∗∗∗*^	0.4585^*∗∗∗*^	0.4624^*∗∗∗*^	0.4624^*∗∗∗*^	0.4773^*∗∗∗*^	0.4869^*∗∗∗*^

Mediating variables	GICP							0.2549^*∗∗∗*^				
	GIC								0.277^*∗∗∗*^			
	GID									0.0466^*∗∗∗*^		
	GBD										1.7735^*∗∗∗*^	
	LCMP											0.2139^*∗∗∗*^

Constant term		1.7520^*∗∗∗*^	2.4208^*∗∗∗*^	4.5027^*∗∗∗*^	0.6159^*∗∗∗*^	2.7554^*∗∗∗*^	1.5046^*∗∗∗*^	1.0581^*∗∗∗*^	0.8342^*∗∗∗*^	1.2948^*∗∗∗*^	0.4123^*∗∗∗*^	0.9153^*∗∗∗*^

Sample size		469	469	469	469	469	469	469	469	469	469	469

*R * ^2^		0.1946	0.2672	0.1680	0.1445	0.1651	0.3233	0.3676	0.3641	0.3668	0.3673	0.3509

*Note.* Significance level: + *P* < 0.10, ^*∗*^*P* < 0.05, ^*∗∗*^*P* < 0.10, and ^*∗∗∗*^*P* < 0.001, which is the same as the full text.

**Table 11:** Moderating effect test 1.

	Coeff	SE	LLCI	ULCI
GICP	0.1998^*∗∗∗*^	0.0411	0.119	0.2805
ER	0.1746^*∗∗∗*^	0.0365	0.0772	0.2206
GICP *∗* ER	0.1489^*∗∗∗*^	0.0365	0.1004	0.2489
*R * ^2^	0.4127			
*R * ^2^-chng	0.0212^*∗∗∗*^			

GICP	0.1888^*∗∗∗*^	0.0417	0.1069	0.2707
FES	0.1679^*∗∗∗*^	0.0385	0.0922	0.2436
GRCP *∗* FES	0.0633	0.0375	−0.0104	0.137
*R * ^2^	0.3949			
*R * ^2^-chng	0.0037			

**Table 12:** Moderating effect test 2.

	Coeff	SE	LLCI	ULCI
GIC	0.2121^*∗∗∗*^	0.0419	0.1297	0.2945
ER	0.1625^*∗∗∗*^	0.0367	0.0903	0.2347
GIC *∗* ER	0.1920^*∗∗∗*^	0.0355	0.1222	0.2619
*R * ^2^	0.4282			
*R * ^2^-chng	0.0361			

GIC	0.2015^*∗∗∗*^	0.0432	0.1166	0.2864
FES	0.1756^*∗∗∗*^	0.038	0.101	0.2502
GIC *∗* FES	0.0433	0.0375	−0.0305	0.1170
*R * ^2^	0.3935			
*R * ^2^-chng	0.0017			

**Table 13:** Moderating effect test 3.

	Coeff	SE	LLCI	ULCI
GID	0.2028^*∗∗∗*^	0.0387	0.1267	0.2789
ER	0.1941^*∗∗∗*^	0.0357	0.1239	0.2643
GID *∗* ER	0.1869^*∗∗∗*^	0.0350	0.1181	0.2556
*R * ^2^	0.4394			
*R * ^2^-chng	0.0346^*∗∗∗*^			

GID	0.2420^*∗∗∗*^	0.0396	0.1641	0.3199
FES	0.2230^*∗∗∗*^	0.0368	0.1508	0.2953
GID *∗* FES	0.0005	0.0363	−0.0708	0.0718
*R * ^2^	0.4115			
*R * ^2^-chng	0.0000			

**Table 14:** Moderating effect test 4.

	Coeff	SE	LLCI	ULCI
GBD	0.2402^*∗∗∗*^	0.0376	0.1497	0.2976
ER	0.2067^*∗∗∗*^	0.0356	0.1368	0.2767
GBD *∗* ER	0.1970^*∗∗∗*^	0.0369	0.1245	0.2695
*R * ^2^	0.4413			
*R * ^2^-chng	0.0339^*∗∗∗*^			

GBD	0.2545^*∗∗∗*^	0.0386	0.1786	0.3303
FES	0.2159^*∗∗∗*^	0.0365	0.1442	0.2875
GBD *∗* FES	0.0263	0.0353	−0.0431	0.0957
*R * ^2^	0.4192			
*R * ^2^-chng	0.0007			

**Table 15:** Moderating effect test 5.

	Coeff	SE	LLCI	ULCI
LCMP	0.1440^*∗∗∗*^	0.0394	0.6650	0.2215
ER	0.1852^*∗∗∗*^	0.0369	0.1128	0.2577
LCMP *∗* ER	0.2044^*∗∗∗*^	0.0364	0.1329	0.2759
*R * ^2^	0.4211			
*R * ^2^-chng	0.0396^*∗∗∗*^			

LCMP	0.1436^*∗∗∗*^	0.0411	0.0629	0.2243
FES	0.1794^*∗∗∗*^	0.0385	0.1038	0.2551
LCMP *∗* FES	0.0690	0.0388	−0.0073	0.1454
*R * ^2^	0.3837			
*R * ^2^-chng	0.0042			

**Table 16:** Moderated mediation effect test 1.

DS ⟶ GICP ⟶ EP				
ER	Effect	Boot SE	Boot LLCI	Boot ULCI
−1	0.0205	0.0277	−0.0268	0.0642
0	0.0806	0.0195	0.0449	0.123
1	0.1407	0.0311	0.0506	0.2012
Intergroup differences	0.1201	0.0380	0.0441	0.1822

Index of moderated mediation				
ER	0.0601	0.019	0.0253	0.1006

**Table 17:** Moderated mediation effect test 2.

DS ⟶ GIC ⟶ EP				
ER	Effect	Boot SE	Boot LLCI	Boot ULCI
−1	0.0093	0.0258	−0.0422	0.0599
0	0.0981	0.0224	0.056	0.1449
1	0.1868	0.0336	0.1259	0.2589
Intergroup differences	0.1776	0.0397	0.1027	0.2568

*Index of moderated mediation*				
ER	0.0888	0.0198	0.0514	0.1284

**Table 18:** Moderated mediation effect test 3.

DS ⟶ GID ⟶ EP				
ER	Effect	Boot SE	Boot LLCI	Boot ULCI
−1	0.0066	0.0239	−0.0407	0.0531
0	0.0845	0.017	0.0521	0.1188
1	0.1624	0.025	0.1161	0.2142
Intergroup differences	0.1558	0.0352	0.0901	0.2287

*Index of moderated mediation*				
ER	0.0779	0.0176	0.0451	0.1144

**Table 19:** Moderated mediation effect test 4.

DS ⟶ GBD ⟶ EP				
ER	Effect	Boot SE	Boot LLCI	Boot ULCI
−1	0.0152	0.020	−0.025	0.054
0	0.0846	0.0182	0.0501	0.1231
1	0.154	0.0285	0.0999	0.2135
Intergroup differences	0.1388	0.0332	0.0788	0.2081

*Index of moderated mediation*				
ER	0.0694	0.0166	0.0394	0.1040

**Table 20:** Moderated mediation effect test 5.

DS ⟶ LCMP ⟶ EP				
ER	Effect	Boot SE	Boot LLCI	Boot ULCI
−1	−0.0218	0.0208	−0.0634	0.0185
0	0.0519	0.017	0.0203	0.0876
1	0.1257	0.0271	0.0767	0.1817
Intergroup differences	0.1474	0.0342	0.0839	0.2180

*Index of moderated mediation*				
ER	0.0737	0.0171	0.0419	0.1090

## Data Availability

The datasets used and/or analyzed during the current study are available from the corresponding author on reasonable request.
